RETRACTED

# A Prospective Evaluation of the Awareness, Knowledge, and Management of Osteoporosis in a Cohort of Medical Staff

**DOI:** 10.1155/2022/4201180

**Published:** 2022-05-28

**Authors:** Xiaoling Zhou, Xin Li, Tingting Wei, Ying Xu, Yuanyuan Mao, Chen Lei

**Affiliations:** ^1^Department of Nephrology, General Hospital of Ningxia Medical University, Yinchuan, Ningxia 750004, China; ^2^General Hospital of Ningxia Medical University, Yinchuan, Ningxia 750004, China; ^3^Department of Geriatrics and Special Needs, General Hospital of Ningxia Medical University, Yinchuan, Ningxia 750004, China

## Abstract

**Objective:**

To investigate the differences in the awareness, knowledge, and management of osteoporosis from a cohort of medical staff after educational intervention.

**Methods:**

A total of 653 medical workers from different departments related to the prevention and treatment of osteoporosis from 7 hospitals in Ningxia were enrolled. Information was collected using a designed questionnaire.

**Results:**

After 5 years of educational intervention and follow-up, medical staff had an increased understanding of osteoporosis diagnosis, including dual-energy X-ray, ultrasound bone sonometer, fragility fracture history, biochemistry markers, and the awareness of the susceptible population. However, there was no improvement in the cognition of single/dual photo absorptiometry, symptoms and signs, and bone turnover index. Their understanding of antiosteoporosis drugs, especially the application of calcitonin, diphosphates, and vitamin D, was significantly promoted, while the perception of indicators and time in follow-up, some adverse drug reactions, and exercise therapy remained unchanged. Medical staff were remarkably less aware of the management of follow-up for osteoporosis, exercise and diet therapy, and bone turnover markers.

**Conclusion:**

A great gap was identified in the perception of osteoporosis among medical staff in the Ningxia region. After the educational intervention, the knowledge regarding some aspects of osteoporosis generally improved. Much more effort should be made to strengthen the training and learning on the special detection methods of osteoporosis, medications and exercise therapy, and follow-up management.

## 1. Introduction

Osteoporosis (OP) is a metabolic skeletal disease characterized by low bone mass, structural deterioration of bone tissue, and increased bone fragility predisposing to an increased risk of fracture, affecting almost one in two older women and one in three older men [1]. With the progress of population aging, the prevalence of OP has increased worldwide, presenting a major source of morbidity and mortality in the elderly and laying a socioeconomic burden throughout the world [2]. Previous epidemiological study has reported that the prevalence of OP in people over 50 years old in industrialized countries ranges from 9% to 38% in women and 1% to 8% in men [3]. It is reported that 25.0% of women and 11.6% of men suffered from OP in Taiwan [4]. Fragility fracture is the most dreadful outcome of OP, leading to a decline in quality of life and an increase in mortality. Besides, once the first fracture occurs, the risk of refracture and premature mortality increases [5].

RETRACTED

OP can be preventable through optimizing peak bone mass, preserving bone mass, and minimizing bone loss at different ages [6]. However, OP still remains an underrecognized and undertreated condition despite the known relationship between OP and fractures. The reported rates of OP diagnosis and its treatment are very low even after hip fracture, ranging from 5–25% [7–9]. Several studies have suggested that active participation of surgeons in the management of OP can be helpful in improving the management of osteoporotic fracture [10–12]. In this setting, an advanced role for physicians in the “front line” of osteoporotic fracture treatment with a better understanding of OP and adequate knowledge of fracture risk is of great importance for preventing subsequent fractures [13].

But, there is a lack of appropriate treatment and management of OP and fragility fractures worldwide. A study has shown that women's experiences of living when they were first diagnosed with OP were related to the treatment of physicians [14]. In the USA, 71.4% of women with OP aged ≥65 did not receive OP treatment, including 75.9% of the subgroup of patients with a prior fracture [15]. Meanwhile, research conducted around the world suggested insufficient knowledge of OP among physicians [16–21].

There have been extensive studies on many potential strategies to prevent OP. Physician education has been viewed as one method of improving awareness and appropriate therapy strategies for OP. In this study, we evaluated the knowledge of OP and the level of OP treatment and management in a medical staff population. In addition, we followed up this cohort for 5 years to determine if there was any change in the perception and management of the population after educational intervention.

## 2. Methods

### 2.1. Populations

This was a prospective cohort study performed in Ning Hui Autonomous Region involving three 3-grade hospitals and four 2-grade hospitals in four cities from 2013-2018. Medical staff in departments related to OP diagnosis and treatment were recruited, including Endocrinology, Orthopedics, Rheumatoloy, Gynecology, Obstetrics, Nephrology, and General Department. All participants voluntarily participated and provided written informed consent after receiving a detailed explanation of the study. This study was approved by the Medical Ethics Committee of the General Hospital of Ningxia Medical University.

RETRACTED

### 2.2. Questionnaire

A total of 700 questionnaires were distributed, and 653 valid questionnaires were collected. This self-designed multiple-choice questionnaire consists of three parts including 15 questions. The first part includes the general information of medical staff (age, gender, department, and professional title). The second part mainly focused on knowledge, diagnosis, bone turnover markers (BTMs), and the application of AODs of OP. The third part was designed to evaluate the follow-up management and other therapies. After 5 years of follow-up, 12 people were dismissed from the cohort due to job transfer. Another 23 people did not give feedback on the questionnaire. The same questionnaire was used to evaluate the results again.

### 2.3. Statistical Analysis

Statistical analyses were performed with SPSS 22.0 software (SPSS, Inc., Chicago, IL, USA). Data were shown as prevalence rates (percent). The chi-square test with Fisher's exact test when necessary was performed to compare the difference in rates. *P* value < 0.05 was considered as statistical significant.

## 3. Results

### 3.1. Assessment of the Basic Knowledge among Participants regarding OP

As is shown in Table 1, the perception rate of the definition, diagnosis, susceptible population, drug types, and follow-up methods of OP was 97.5%, 60%, 36.4%, 10.4%, and 5.8%, respectively, and after education intervention the perception rates were 98.6%, 69.3%, 45.4%, 31.0%, and 7.6%, respectively. We found that the medical staff in Ningxia exhibited the greatest knowledge of the definition of OP and had insufficient knowledge of the types of drugs and diagnostic methods, while had the lowest awareness of vulnerable people and follow-up of OP. After education intervention, the overall knowledge of OP increased, apparently except for the definition (*P* < 0.001).

### 3.2. Evaluation of the Knowledge among Participants regarding Diagnostic Methods and Special Tests

The perception rate regarding the diagnostic methods including dual-energy X-ray (DEXA), single/dual photo absorptiometry (SPA/DPA), ultrasound bone sonometer (UBS), and symptoms and signs and history of fragile fracture were 15.5%, 38.1%, 21.7%, 59.4%, and 33.5%, respectively, and 20.6%, 31.5%, 40.8%, 55.3%, and 59.4% separately after educational intervention (Table 2). As to the special testing methods, only 7.8% of the participants knew the biochemical indicators needed to be tested for OP, 5.2% knew that testing BTMs were needed for OP, and 19.8% knew detecting vitamin D was necessary for OP. After education intervention, the awareness rates were 14.4%, 6.8%, and 72.1%, respectively. In the investigation of various diagnostic methods, doctors and nurses were knowledgeable about symptoms and signs, but their knowledge of DEXA, SPA/DPA, UBS, and history of brittle fracture is obviously low. After education intervention, their awareness of SPA/DPA, UBS, and osteoporotic fracture history also remarkably increased (*P* < 0.05), yet it was discouraging that the overall state of cognition was still pessimistically low. Medical staff were almost knowledgeable about special detection methods for OP, among which the recognition of bone turnover indicators is the lowest and has not been improved after educational intervention. Educational intervention had a surprising impact on the cognition of vitamin D. The cognitive rate increased from 19.8% to 72.1% (*P* < 0.001), and the cognition of biochemical indicators also improved significantly (*P* < 0.001).

RETRACTED

### 3.3. Investigation of the Knowledge among Participants regarding Follow-Up and Nondrug Therapy

Only 2.1% and 3.4% of the participants knew about the indicators and follow-up time of OP (Table 3). It was shocking that only 0.6% of the participants knew about exercise and dietary therapy. After education intervention, only the cognitive rate of dietary therapy was improved (*P* < 0.01), while the other cognitive levels were not different. Medical staff had a great lack of knowledge about follow-up of OP. They hardly know about exercise and diet therapy. After educational intervention, they had evidently improved their knowledge of diet therapy.

### 3.4. Assessment of the Basic Knowledge among Participants regarding Medication

Compared with the perception rate of 99.7% on calcium and 42.1% on vitamin D, only 9.8% and 2.1% of participants had an understanding about calcitonin and bisphosphate, while merely 8.1%, 2.9%, and 5.1% knew about the side effects of calcitonin, oral administration, and intravenous bisphosphonate.

In the investigation of anti-OP drugs, we found that medical staff had a higher awareness of calcium supplements, but a lower awareness of the application of calcitonin and bisphosphonate. However, after education intervention, the awareness of both was significantly improved (9.8% vs. 14.0%, *P* < 0.01; 2.1% vs.14.7%, *P* < 0.01). There was also a significant lack of awareness of adverse drug reactions of anti-OP drugs among medical staff. The awareness of the side effects of calcitonin drugs increased sharply after educational intervention (8.1% vs. 15.8%, *P* < 0.01) as well as oral bisphosphonate (2.9% vs. 9.4%, *P* < 0.01). There was no change in intravenous bisphosphonate (Table 4).

RETRACTED

## 4. Discussion

There are many factors influencing the enthusiasm of doctors for the prevention and treatment of OP. Most doctors and nurses thought OP was out of their major specialty, and the lack of enough knowledge and experience made it harder for them to study. A few people thought that OP was not valued and recognized, and it was difficult to learn and had low benefits, while a few were not interested at all. In Ningxia, many diagnostic techniques and laboratory examinations for OP have not been fully popular, especially in primary hospitals, where doctors have fewer patients with OP and lack of experience. Meanwhile, the limitation of dosage forms and application scope of anti-OP drugs and their high prices both restrict clinical use. The national medical insurance policy also makes many new drugs temporarily unable to enter the clinic, hindering the recognition of medical workers. In this study, we found that medical staff in Ningxia have an obvious lack of knowledge regarding diagnostic methods, BTMs, follow-up, and OP medications. This result was also consistent with the other two studies [22, 23]. In addition, remarkable gaps were revealed in understanding regarding AOPs, adverse effects of medications and diet and exercise medications. As shown, physicians exhibited much less knowledge about the side effects of the anti-OP drugs and other medications, which is similar to the findings of another study in Israel [23].

We are gratified that, after the intervention of education and learning, medical workers are much more knowledgeable about OP, especially in the diagnosis of OP, the indicator to detect vitamin D, and the application of calcitonin and bisphosphonate. Comparative studies focused on interventions for improving OP management demonstrated that awareness of orthopedic surgeons had a greater effect on OP management rates after hip fracture [11, 24]. Kim et al. conducted a prospective study and found an improved medication rate of OP from 15% to 32% after 2 years of education to orthopedic surgeons [25]. However, even after the educational program, the state of medical staff's cognition on bone turnover indicators, follow-up management and other therapies remained unchanged. Another study has shown that after 1-year educational program, the rate of calcium and vitamin D and bisphosphonate prescriptions increased notably while the follow-up evaluations did not differ [26]. This result indirectly confirmed our investigation, suggesting that there are shortcomings in the follow-up and treatment management of OP. The improvement of orthopedic surgeons' awareness of the importance of identifying patients with OP has proved beneficial [27]. More effective educational programs of OP treatment and targeted learning plans should be warranted and great efforts should be emphasized at the political and administrative levels.

RETRACTED

The limitations of this study should be acknowledged. This survey is mainly aimed at the postosteoporotic fracture management survey. Orthopedic and general doctors accounted for a higher proportion of participants, while the number of other departments participating in the survey was relatively limited, which may have led to deviations in the results. In addition, this study preliminarily investigated the theoretical knowledge of OP among doctors and nurses, and the questionnaire did not involve doctors' clinical treatment of OP. A longitudinal study with a repeated measure design is needed to observe whether the changes in knowledge could have a significant impact on clinical OP practice management.

## 5. Conclusions

This study indicated that a significant lack was identified in knowledge and awareness pertaining to OP in Ningxia. Education intervention can be effective in promoting part of cognition. It is indispensable for escalating the efforts to give more attention to medical education and improve the knowledge of medical workers regarding various aspects of OP management.

## Figures and Tables

**Table 1:** Basic knowledge among participants regarding osteoporosis.

		Definition	Diagnosis	Susceptible people	AOPs	Follow-up
Pre-edu	*N*	637	392	238	68	38
	Percent	97.5%	60%	36.4%	10.4%	5.8%
After-edu	*N*	699	491	322	220	54
	Percent	98.6%	69.3%	45.4%	31.0%	7.6%
*χ* ^2^		1.963	12.679	11.294	86.647	1.743
*P* value		0.161	0.000	0.001	0.000	0.187

Pre-edu: pre-education; after-edu: after education; AOPs: antiosteoporosis drugs. *P* < 0.05 is statistically significant.

**Table 2:** Perception among participants regarding diagnostic methods and special tests.

		Diagnostic methods					Special tests		
		DEXA	SPA DPA	QUS	Symptoms and signs	Fragile fracture history	Biochemical indicators	Vit D	BTMs
Pre-edu	*N*	101	249	142	388	219	51	129	34
	Percent	15.5%	38.1%	21.7%	59.4%	33.5%	7.8%	19.8%	5.2%
After-edu	*N*	146	223	289	392	421	102	511	48
	Percent	20.60%	37.50%	40.80%	55.30%	59.40%	14.4%	72.1%	6.8%
*χ* ^2^		6.015	1.696	56.825	2.368	91.131	14.743	373.532	1.468
*P* value		0.014	0.080	0.000	0.124	≤0.001	≤0.001	≤0.001	0.226

Pre-edu: pre-education; after-edu: after education; DEXA: dual-energy X-ray; SPA/DPA: single/dual photo absorptiometry; UBS: ultrasound bone sonometer; BTMs: bone turnover markers; Vit D: vitamin D. *P* < 0.05 is statistically significant.

RETRACTED

**Table 3:** Knowledge among participants regarding follow-up and nondrug therapy.

		Follow-up indicators	Follow-up time	Exercise therapy	Diet therapy
Pre-edu	*N*	14	22	4	4
	Percent	2.1%	3.4%	0.6%	0.6%
After-edu	*N*	25	28	12	18
	Percent	3.5%	3.9%	1.7%	2.5%
*χ* ^2^		2.335	0.324	3.415	7.936
*P* value		0.127	0.569	0.065	0.005

Pre-edu: pre-education; after-edu: after education. *P* < 0.05 is statistically significant.

**Table 4:** Basic understanding among participants regarding medication.

		Application				Adverse effects		
						Bisphosphate		
		Calcium	Vit D	Calcitonin	Bisphosphate	Calcium	Oral	Intravenous injection
Pre-edu	*N*	651	275	64	14	53	19	33
	Percent	99.7%	42.1%	9.8%	2.1%	8.1%	2.9%	5.1%
After-edu	*N*	675	412	88	104	27	24	37
	Percent	95.2%	58.1%	14.0%	14.7%	15.8%	9.4%	5.2%
*χ* ^2^		26.621	34.797	25.439	67.385	19.412	17.251	0.019
*P* value		≤0.001	≤0.001	≤0.001	≤0.001	0.001	0.006	0.890

Vit D: vitamin D. *P* < 0.05 is statistically significant.

## Data Availability

The data used to support the findings of this study are available from the corresponding author upon request.
